RETRACTED

# Interactive Music Learning Model Based on RBF Algorithm

**DOI:** 10.1155/2022/5759986

**Published:** 2022-08-13

**Authors:** Fengqin Liu

**Affiliations:** Fujian Institute of Education, Fuzhou 350001, Fujian Province, China

## Abstract

With the development of art education and information technology, it is increasingly necessary to use computer technology and multimedia technology to assist teaching in the teaching activities of music subjects nowadays, so as to cultivate students' independent inquiry ability and drilling ability. The design of an interactive teaching music intelligence system based on artificial intelligence is studied, and a music learning model based on the RBF algorithm is proposed, which helps to enhance students' inquiry ability and also plays the leading role of teachers. By teaching each other, students become the main subject of teaching and learning, and it stimulates students' enthusiasm and learning awareness of music learning.

## 1. Introduction

Artificial intelligence technology originated in the 1950s [1]. Artificial intelligence is a theory, method, technology, and application system that uses digital computers or machines controlled by digital computers to simulate, extend, and expand human intelligence, perceive the environment, acquire knowledge, and use the knowledge to obtain the best results. The era of artificial intelligence has arrived and will further assist human analysis and decision-making, reform human work patterns, and even replace some human work in the future. In the late twentieth century, along with the rapid development of science and technology, music classrooms accepted and applied more efficient, intelligent, and humanized synthetic musical instruments, and the renewal of these instruments showed more convenient, intelligent and perfect characteristics [2–4]. The application of scientific and technological tools in the field of music has laid the foundation for the creation of new works, while providing music educators with new directions and pedagogical thinking. Now, in the age of artificial intelligence and big data, how should the role of music teachers be transformed to promote the development of music education? How can teachers use AI technology in music education to improve our teaching? How can music teachers be empowered to fully reflect the value of music teachers? This paper proposes an interactive music learning mode based on the RBF algorithm, which provides some reference for the efficient development of music classroom teaching.

## 2. Development of Artificial Intelligence

### 2.1. Research on Artificial Intelligence in Music Education

The combination of artificial intelligence and music has existed for quite a long time. Since the International Computer Music Conference held in the United States in 1974, the development of digital sound processing and software programs for music has come a long way, and the combination of artificial intelligence and music education has produced numerous research results [5, 6]. The Tonara app, currently developed by the Israeli technology education company Tonara, is the first interactive sheet music app on the iPad. Based on the development of artificial intelligence, the Tonara app can follow the beat and rhythm of the player to achieve automatic page turning, providing sheet music for five instruments, which can be used as a supplementary tool for musicians to practice. The interactive music platform Wolfie, launched later, uses AI technology combined with a music database to provide an objective evaluation tool for classroom or student performance music and error correction, covering a variety of music styles such as jazz and rock. In order to achieve an all-in-one interactive way of teaching musical instruments and intelligent mobile terminals, gamified pianos such as Theone have emerged and reduced the degree of human intervention, using the assistance of multimedia, towards emotional robotics and deep learning, making the efficiency of learning and practicing greatly increased, which contains a model of the pedagogue and a model of the learner, embodying the entire content of the development of the teaching system and feedback to learners in time to form a good teaching loop.

RETRACTED

### 2.2. Emotional Machines and Emotional Interaction Theory

Emotion is a special way of thinking for human beings, containing complex operating mechanisms, and it is used to develop the technical challenges of artificial intelligence by shaping machines to acquire emotions, mainly through the creation of six dimensions of emotional machines applied to music teaching. The six dimensions given by Marvin Minsky, the “father of artificial intelligence,” are “consciousness,” “mental activity,” “common sense,” “thinking,” “intelligence,” and “self.” These six dimensions explain the complex mechanisms of the human brain, and thus confirm the possibility of applying emotional machines to music teaching [7]. Emotional interaction is an artificial intelligence-based emotional computing proposed by Prof. Picard of MiT Media Lab. Emotional computing is the process of giving computers or machines the ability to observe, understand, and perform various emotions similar to or the same as human communication. Emotional interaction is a hot research direction in the field of artificial intelligence, aiming to make the process of communicating with machines or computers more natural and convenient [8–10]. For personalized music education, AI teachers similar to Siri exist to solve students' problems when they encounter them, and when there is an error in music practice, the intelligent system talks about this error, as shown in Figure 1.

RETRACTED

Music knowledge learners access the learning combination, generally the learning platform, by logging into the client and then presenting the learning results to the instructor through the human-computer interaction mode. The instructor, in turn, refines the new lecture model and teaching model through the results to improve the learners' learning awareness and learning ability based on negative feedback, forming a perfect interactive closed loop. Compared with traditional assessment methods, the AI-based teaching system uses developmental feedback and rational application of emotional evaluation to enhance the teaching efficiency of music learners.

## 3. Music Intelligent System Analysis and Implementation

The core algorithm model of the interactive teaching music intelligence system uses the artificial intelligence algorithm—RBF algorithm. This algorithm, called radial basis function, is a neural network composed of locally tuned neurons and generally has a five-layer network model, as shown in Figure 2.

The first layer is the case-related information factors, and these inputs can be grouped into different music item metrics that are fed into the neural network structure. The second layer is the affiliation function with a mathematical expression, as in (1) [9]:

(1) $$\begin{array}{c} \mu_{ij}\left(x_{i}\right)=\exp\left[\frac{{\left(x_{i}-c_{ij}\right)}^{2}}{\sigma_{j}^{2}}\right],i=1,2,\ldots r;\;j=1,2,\ldots ,u. \end{array}$$

The third layer describes the number of fuzzy rules, which are learned by the samples, trying to make the least number of rules learned and the most important. The mathematical calculation of the output of the *j*th of these rules is shown in (2) [10, 11]:

(2) $$\begin{array}{c} \phi_{j}=\exp\left[-\frac{\sum_{i=1}^{r}{\left(x_{i}-c_{ij}\right)}^{2}}{\sigma_{j}^{2}}\right]=\exp\left[-\frac{{\left\|X-C_{j}\right\|}^{2}}{\sigma_{j}^{2}}\right],j=1,2,\ldots ,u, \end{array}$$

where *C*_*j*_=(*c*_*j*_,…, *c*_*rj*_) denotes the center of the *j*th R_B_F unit. The RBF neural network is characterized by the fact that the closer the neuron is to the center, the higher its activation, which is very much in line with the teaching model of the influencing factors of interactive music learning.

The fourth layer is the normalization layer, and the nodes of this layer should be consistent with the fuzzy rule nodes, and the output of its *j*th node is as shown in (3) [11]:

(3) $$\begin{array}{c} \psi_{j}=\frac{\phi_{j}}{\sum_{k=1}^{N}\phi_{k}},j=1,2,\ldots ,u. \end{array}$$

The fifth layer is the output layer, which outputs the evaluation of each skill of music performance, and its output, which is mainly based on the TS fuzzy model in the RBF algorithm, is as shown in (4):

(4) $$\begin{array}{c} y\left(x\right)=\frac{\sum_{i=1}^{u}\left[\left(a_{i0}+a_{i1}x_{1}+\ldots +a_{1r}x_{r}\right)\exp\left(-{\left\|x-c\right\|}^{2}/\sigma_{i}^{2}\right)\right]}{\sum_{i=1}^{u}\exp\left(-{\left\|x-c_{i}\right\|}^{2}/\sigma_{i}^{2}\right)}, \end{array}$$

where *ω*_*k*_ is the connection representing the *k*th rule, i.e., the summation of the weight products of the output variables, as in (5).

(5) $$\begin{array}{c} y\left(x\right)=\sum_{k=1}^{u}\omega_{k}\cdot \psi_{k}. \end{array}$$

The interactive music learning model based on the RBF algorithm is to incorporate the algorithm concept in the design of the platform and to fully present the algorithm when writing the code, and to implement it in the functionality of the platform interface so that it effectively fits into the interactive learning model [12–14]. *X* is the proportion of learning time consumed in the interactive music intelligence system by 100 students selected from all surveyed students who passed the music test with excellent performance; *c*_*j*_*σ*_*j*_ is the distribution of the implied layers of each music learning courseware for the corresponding term (*x*) learning time for students with excellent performance, and the implied layer categories of these learning samples are relatively parallel; *y* is the optimal music performance corresponding to each input layer. To achieve simplification of the RBF algorithm, the second, third, and fourth layers can be grouped into implicit layers, and the first and fifth layers are the input and output layers, respectively, for different aspects of music teaching as the input layers of the algorithm [15]. When targeting a series of larger scale data, the first *M* data of music data are used as the initial training, and then the RBF model of students' learning music knowledge is constructed, which is continuously evaluated by the designed software platform until the perfect model is finally constructed. Its program design diagram is shown in Figure 3.

RETRACTED

## 4. Strategies Related to the Interactive Music Learning Model

### 4.1. Using Music Classroom Activities to Create an Interactive Learning Platform

“Interactive” learning refers to the reasonable use of various teaching methods (multimedia network technology and online resources) in teaching activities to form a cooperative relationship of communication and interaction between teachers and students, so that students can complete the transformation from “learning” to “learning,” “good learning” to “will learn” “learn” transformation [16]. The core of activity teaching is “activity,” and the practicality of the content and the main activities of the students must be clear. The teaching process is really based on students' independent activities and active exploration, and through students' comprehensive and diversified main practical activities, it promotes the overall development of their subject spirit, practical ability, and various qualities. It should be said that the combination of interactive teaching and activity teaching methods is a new form of education and teaching, but also a kind of education and teaching ideas and thoughts [17].

With the use of smart classrooms (multimedia classrooms) in schools at this stage, teachers can actively use network resources to create teaching activities. For example, the appreciation lesson “A Guide to Youth Orchestras” is an orchestral piece written by British composer Benjamin Britten in 1946 for the British government's educational film “Instruments of the Orchestra.” The theme of the piece is taken from Henry Purcell's dramatic score for the play Revenge of the Moor, and a series of variations on this theme introduce the various instruments in the orchestra. During the actual lesson, with the powerful sound equipment function of the Smart Classroom, students can conduct active listening and identification activities in conjunction with the classification of orchestral instruments, and feel the difference between woodwind, brass, string, and percussion instrument groups from the music. And after the instrument grouping is confirmed to further listen to and identify the sound effects of different instruments, students practice completing their learning tasks through verbal descriptions, humming, and imitating activities, which is an effective role of interactive learning platform construction. At the same time, combined with classroom teaching design, teachers can also actively use online resources in the classroom to pack other pieces played by different instruments in a unified way, and students can carry out self-hearing and self-discussion learning under the guidance of the teacher, and complete the differentiation of instrument types with the help of corresponding effective teaching activities [18]. Of course, after the class, we intentionally arrange students who have the foundation of playing instruments to practice creating harmonies, or to practice ensembles of different instrument groups, which is also an extension of classroom teaching and learning; moreover, it can cultivate students' creative ability and cooperation ability, and motivate them to go farther and farther on the road of music.

RETRACTED

### 4.2. Using Classroom Groups to Help Each Other and Create an Interactive Learning Situation

Interactive group learning is an important form of interactive learning, which is a kind of teaching and learning activity carried out by group activities. Teachers are required to purposefully divide the class into groups according to “intergroup homogeneity, intra-group heterogeneity” or “intergroup heterogeneity, intra-group homogeneity” before the lesson, so that each group has a strong cohesive force, and at the same time, each group is not isolated from each other, and teachers must promote intergroup interaction in order to truly open up a new pattern of classroom learning, avoiding problems such as students only listening but not remembering, learning but not thinking, and avoiding letting the questioning always hide in the shadows of knowledge, and bringing students into a more dazzling stage. In the teaching design process, the teaching links are required to highlight group activities as the core, requiring students to cooperate with each other to try to explore knowledge, which helps students to stimulate their interest in learning, and is conducive to students of different levels to play the initiative of learning in the time and space created, which plays an active role in the cultivation of students' thinking and optimizing the cooperation between teachers and students. At the same time, in the classroom teaching fascinating contextual design (problem design) can also attract students' eyes and inspire students' thinking, for teaching the icing on the cake. In this way, the means of creating learning contexts and stimulating effective individual and group learning behaviors are particularly important [19]. Interactive whiteboards can fill the teaching gap due to their visual, interactive and generative advantages.

In the actual lesson, teachers can combine the learning situation with grouping activities according to the grouping principles mentioned above. Also combined with the characteristics of subject teaching, interactive whiteboards can also be used to integrate and implement subject knowledge with outstanding compatible effects. For example, when teaching “The Language of Drums,” teachers can use the electronic whiteboard to show students African drums, as the representative musical instrument of West African Manding culture, which gives a refreshing feeling from appearance to timbre [20]. Students can analyze and learn about the instrument through group guesses, listening and recognition quizzes, and visual discussions with the help of the work “Dance of Fondom Fromm.” In addition, the interactive whiteboard enables teachers to create vivid images for students through language, music, and video playback. In addition, the use of interactive whiteboard also enables teachers to create vivid scenes for students through verbal depiction, musical rendering, and video playback, combining the abstract nature of subject knowledge and the image of students' thinking, thus optimizing teaching and enhancing teaching effects. For example, the title song of “Animal World” composed by the French band Space is full of dynamic and fantasy music, beautiful electronic sound effects, and spirited movement melody combined with the video all stir up strong resonance for the listener. When students use this context to study in groups, according to the teacher's question design and prompting guidance, the learning atmosphere will become more and more intense, and the discussion can also develop a rich imagination, the classroom effect is positive and effective.

RETRACTED

### 4.3. Using the Classroom Composition Process to Develop Interactive Learning Habits

Music composition teaching is a teaching activity that uses various music materials for music learning in order to cultivate and develop students' creative spirit and creative ability [21, 22]. In the teaching process, teachers should create lively and interesting activities according to the teaching objectives, so that students can participate in creation and experience creation, thus achieving the purpose of mastering certain music knowledge and skills and further gaining the emotional experience of music. Because of the limited musical foundation and ability of students, teaching should focus on promoting the harmonious generation and dynamic development of students' creative enthusiasm, desire for knowledge, feeling experience, and aesthetic expression.

In our study of music teaching theories, we also found that the Dacroix Method has a very distinct statement for the elaboration of improvisation lessons: students are able to complete improvisation activities and performances in the process of being educated. Likewise, the rhythmic solitaire and rhythmic-melodic quiz in the Kodály method makes a strong statement about the learning space and effectiveness of the music classroom. The Orff teaching method affirms the concept of active and creative music teaching and believes that students' learning and creation process is divided into four stages: exploration, imitation, improvisation, and creation, which is a kind of music education aiming at inspiring people's imagination and developing their creative potential [23, 24]. In the actual teaching, in view of the psychological and physiological characteristics of junior high school students, it is necessary to make use of the network interactive resources and adopt a step-by-step process to advance gradually, suggesting the implementation of melody modeling and rhythm discrimination in grade 7: through classroom teaching methods and practical demonstrations, train students to model melody singing within 4–8 bars and be able to identify rhythm types, which can be extended to rhythm imitation and creation. Creative “bridging” can also be done: that is, it can be effectively implemented in a variety of music teaching activities. Examples include setting poems to music, filling in the blanks with musical phrases, reflecting melodies, and improvising lyrics. In the eighth and ninth grades, students will practice their basic compositional skills, and through pedagogical guidance and practical application, they will be able to improvise 4–8 bars or complete short compositions (marches, minuets, tangoes, etc.) in predetermined contexts. Of course, in interactive learning, thanks to the digital teaching features: the use of ipad music software and accompaniment, the integration of Dalcroze's body rhythms to increase the fun of music lessons; the use of Kodály's “Corvin gestures” to build the children's concept of pitch; the use of Orff's music-language. The use of Orff's music-verbal-movement triad allows students to improvise and engage in activities that get the class moving.

RETRACTED

### 4.4. Enriching Interactive Learning Outcomes by Using In-School and Out-of-School Club Curriculum Activities

#### 4.4.1. Leveraging School Art Clubs to Foster Regular Learning inside and outside the Classroom

Learning within the classroom lays a good foundation for students to learn. Using school art clubs interactively after school can be effective in further enriching creative outcomes [25]. Street dance club combinations, choral club practices, band collaborations, etc. can actively create a space where students enjoy interacting. At the same time, teachers should also make use of school cultural and art festivals, community gala, and art shows to boost students' self-confidence and desire to express themselves, which in turn brings out the children's learning outcomes.

#### 4.4.2. Using Network Resources for Effective Choreography Activities

Music teachers should actively communicate with the IT subject teachers to break the disciplinary boundaries and allocate corresponding music teaching network resources in the school computer room in due course, and develop and implement them as school-based courses. Classroom learning and practice results can also be displayed on the platform, trying to use the network platform for correction [26]. Students can also make use of the music network teaching resources to make adaptations or compositions through interactive learning.

RETRACTED

#### 4.4.3. Encourage Students to Dare to Create through Learning Assessment

Composing music is a very effective means of arousing students' motivation to learn music. In the process of learning to compose, students must inevitably relate their musical knowledge such as rhythm, beat, melody, and key as well as skills and techniques such as reading music, notation, singing, and playing instruments, and express their inner world with the help of the above means, so as to complete the practical practice of their works. For example, most students do not like to learn to read music because they do not need to read music in their daily life. Therefore, teachers need to actively guide students through classroom instruction, use motivating and effective assessments (individual classroom extra credit, group assessment, and music grade percentages), and provide opportunities for students to demonstrate their musical skills in order to create a strong desire to learn creative writing. By constructing an “interactive” learning model, it is clear that students' thinking skills are enhanced and their individual musical perception, participation, confidence, and expression are strengthened [27–35]. In terms of knowledge, experience, personality, spirit, culture, etc., the vision is enhanced, life is empathized and experienced, life is enlightened, and spirituality is enriched, and the direction of development of teachers and students tends to the realm of truth and beauty. What is more crucial is to be able to understand the musical elements with the help of different expressions such as teaching activities, language and network resources, and teachers are able to clearly see the little changes in students, teaching with fun.

## 5. Conclusion

Interactive teaching music intelligence system provides music learners with better technical support and learning concepts. This paper firstly introduces the theoretical basis of artificial intelligence-based music education and the current status of domestic and international research and analyzes the advantages compared with traditional music teaching methods. And analyze the neural network model, especially targeted RBF algorithm for teaching music intelligent system, consider the training model and construction method of neural network, simulate the learning law of music learners, so as to better realize the effect of interactive teaching music intelligent system, let students immerse in the interactive music intelligent system, through the evaluation of music intelligent system design, can better make improvements to the software design. In the subsequent research, a more humanized interface design should be added, and a larger scale model sample should be used to realize artificial intelligence to make the accuracy more universal and ensure a good stability in terms of operation degree, and also a variety of artificial intelligence algorithms can be fused to improve the training algorithm of neural networks to obtain a more general music intelligence system, which is the key direction of the next research.

RETRACTED

## Figures and Tables

**Figure 1:** Emotional interaction relationship.

**Figure 2:** Structure diagram of the R B F algorithm.

**Figure 3:** Programming drawing.

## Data Availability

The dataset can be accessed upon request.

## References

[1] Wang X. New wind direction of future music: artificial intelligence to empower music development - review of the World Music Artificial Intelligence Conference. *People’s Music*.

[2] Wenhui (2021). Reflections on the interaction between artificial intelligence technology and music education. *Sichuan drama*.

[3] Shen J. (2021). Research on innovation of college music teaching based on artificial intelligence technology. *Food Research and Development*.

[4] Tong X. Na, Yang Q. (2021). The change and response of music communication in the era of artificial intelligence. *Media*.

[5] Pei G., Li T., Wang Y. (2021). Innovative development of music therapy in the era of artificial intelligence. *Zhangjiang Science and Technology Review*.

[6] Zhang J., Zhao Y. (2021). Research and application of interactive teaching music intelligence system based on artificial intelligence. *Microcomputer Applications*.

[7] Chen Y., Zhang K., Liu L. (2021). The “musical personality” of artificial intelligence music--giving dynamicity to music creation to enhance the emotionality of music. *China Ethnic Expo*.

[8] Xiao Ke (2021). Into deep learning, innovative teaching practice - a practical study on the integration of artificial intelligence technology and elementary school music teaching. *Art Review*.

[9] Wang Z. (2020). Research on the application of artificial intelligence in music and its development strategy. *Northern Music*.

[10] Liu H., Han B. (2020). The current situation and challenges of the development of artificial intelligence music. *People’s Music*.

[11] Pan W. (2020). The situation and response of music teaching in colleges and universities in the era of artificial intelligence--Taking the teaching of sight singing and ear training as an example[J]. *Education in Science*.

RETRACTED

[12] Chen S. Z. (2020). An introduction to the application of artificial intelligence technology in music composition. *Music Exploration*.

[13] Wang X., Lei Q. (2019). The penetration and innovation of artificial intelligence on China’s music industry chain. *Modern Communication*.

[14] Liu H. (2019). Artificial intelligence and computer composition:premises, techniques and problems. *Music in Art*.

[15] Yuan Q. (2019). Research on the application of artificial intelligence in music education. *Northern Music*.

[16] Yewen C., Guo W. (2019). Research on the application of artificial intelligence system in the teaching of music education in primary and secondary schools. *Art Review*.

[17] Li W. Y., Zhao T. T., Xu H. M. (2019). The role of EGFR mutation as a prognostic factor in survival after diagnosis of brain metastasis in non-small cell lung cancer: a systematic review and meta-analysis. *BMC Cancer*.

[18] Cao M., Guo W. (2019). Exploring the application value of artificial intelligence system in music education in primary and secondary schools. *Northern Music*.

[19] Chen G. (2019). A popular science course on “music and artificial intelligence” for graduate students in music and art schools. *Computer Education*.

[20] Wang H., Jiao W. (2019). Research on fingerprint retrieval technology of music fragments based on artificial intelligence recognition. *Automation and Instrumentation*.

[21] Sun D. (2019). How primary and secondary school music teachers cope with the arrival of the era of artificial intelligence. *Northern Music*.

[22] Liang X., Li Z. (2019). The interdisciplinary dialogue between music and computer--Side note of the 2018 workshop on the development of artificial intelligence in music. *People’s Music*.

[23] Li W., Gao Z. F. (2018). Music information retrieval technology:the integration of music and artificial intelligence. *Artistic exploration*.

[24] Fu X. (2018). Ethical reflection on musical artificial intelligence--”self-regulation” and “other-regulation” of algorithmic composition. *Artistic exploration*.

[25] Zhou Li, Deng Y. (2018). Exploring the current situation and trends of the development of artificial intelligence composition. *Artistic exploration*.

[26] Zou M. (2018). Artificial intelligence and its application in music education. *Northern Music*.

[27] Ren K. (2018). Music catechism and music teaching innovation under the “Internet+” thinking. *Chinese Music*.

[28] Li L., Mao C., Sun H., Yuan Y., Lei B. (2020). Digital twin driven green performance evaluation methodology of intelligent manufacturing: hybrid model based on fuzzy rough-sets AHP, multistage weight synthesis, and PROMETHEE II. *Complexity*.

RETRACTED

[29] Huang Y. (2022). Construction of “interactive” English translation teaching model based on data-driven learning. *Wireless Communications and Mobile Computing*.

[30] Li L., Qu T., Liu Y. (2020). Sustainability assessment of intelligent manufacturing supported by digital twin. *IEEE Access*.

[31] Wang Q., Zhao C., Qiang Y., Zhao Z., Song K., Luo S. (2021). Multitask interactive attention learning model based on hand images for assisting Chinese medicine in predicting myocardial infarction. *Computational and Mathematical Methods in Medicine*.

[32] Li L., Lei B., Mao C. (2022). Digital twin in smart manufacturing. *Journal of Industrial Information Integration*.

[33] Cao F., Cai J. (2022). Online and offline interaction model of international Chinese education based on few-shot learning. *Computational Intelligence and Neuroscience*.

[34] Li L., Mao C. (2020). Big data supported PSS evaluation decision in service-oriented manufacturing. *IEEE Access*.

[35] Yin X., Chen L., Sun Le (2022). A cross-modal image and text retrieval method based on efficient feature extraction and interactive learning CAE. *Scientific Programming*.

